# The Role of Janus Kinase/STAT3 Pathway in Hematologic Malignancies With an Emphasis on Epigenetics

**DOI:** 10.3389/fgene.2021.703883

**Published:** 2021-12-21

**Authors:** Elham Zeinalzadeh, Alexey Valerievich Yumashev, Heshu Sulaiman Rahman, Faroogh Marofi, Navid Shomali, Hossein Samadi Kafil, Saeed Solali, Mehdi Sajjadi-Dokht, Sajjad Vakili-Samiani, Mostafa Jarahian, Majid Farshdousti Hagh

**Affiliations:** ^1^Student Research Committee, Tabriz University of Medical Sciences, Tabriz, Iran; ^2^Hematology and Oncology Research Center, Tabriz University of Medical Sciences, Tabriz, Iran; ^3^Department of Prosthetic Dentistry, Sechenov First Moscow State Medical University, Moscow, Russia; ^4^College of Medicine, University of Sulaimani, Sulaimaniyah, Iraq; ^5^Department of Medical Laboratory Sciences, Komar University of Science and Technology, Sulaimaniyah, Iraq; ^6^Department of Immunology, School of Medicine, Tabriz University of Medical Sciences, Tabriz, Iran; ^7^Immunology Research Center, Tabriz University of Medical Sciences, Tabriz, Iran; ^8^Drug Applied Research Center, Tabriz University of Medical Sciences, Tabriz, Iran; ^9^German Cancer Research Center, Toxicology and Chemotherapy Unit (G401), Heidelberg, Germany

**Keywords:** leukemia, epigenetics, Janus kinase, STAT3, methylation

## Abstract

The Janus kinase (JAK)/signal transducer and activator of transcription (STAT) signaling pathway has been known to be involved in cell growth, cellular differentiation processes development, immune cell survival, and hematopoietic system development. As an important member of the STAT family, STAT3 participates as a major regulator of cellular development and differentiation-associated genes. Prolonged and persistent STAT3 activation has been reported to be associated with tumor cell survival, proliferation, and invasion. Therefore, the JAK-STAT pathway can be a potential target for drug development to treat human cancers, e.g., hematological malignancies. Although STAT3 upregulation has been reported in hematopoietic cancers, protein-level STAT3 mutations have also been reported in invasive leukemias/lymphomas. The principal role of STAT3 in tumor cell growth clarifies the importance of approaches that downregulate this molecule. Epigenetic modifications are a major regulatory mechanism controlling the activity and function of STAT3. So far, several compounds have been developed to target epigenetic regulatory enzymes in blood malignancies. Here, we discuss the current knowledge about STAT3 abnormalities and carcinogenic functions in hematopoietic cancers, novel STAT3 inhibitors, the role of epigenetic mechanisms in STAT3 regulation, and targeted therapies, by focusing on STAT3-related epigenetic modifications.

## Introduction

Signal transducers and activators of transcription (STATs) are a family of seven cytoplasmic transcription factors that receive the signals from cell-surface cytokine receptors and growth factor receptors and transmit them to the cell nucleus (Morris et al., 2018; Hosseini et al., 2020). The STAT proteins participate in normal cellular events, such as survival, proliferation, and differentiation. The signals produced by the Janus kinase (JAK)/STAT signaling pathway are essential to the blood circulatory system and immune response (Murray, 2007). Activation of cytokine receptors induces anti-apoptotic, proliferative, and differentiation signals, determining the development of different blood cell lineages (Hirano et al., 2000; Robb, 2007). Clinical trials have shown that STAT3 is constitutively active in many types of cancer, including breast cancer, hepatocellular carcinoma, multiple myeloma, lymphoma, and prostate cancer. Moreover, the contribution of the mutant JAK2 in myeloproliferative diseases, polycythemia vera, adult T-cell lymphoblastic leukemias, acute lymphoblastic leukemia, and Hodgkin lymphoma (HL) has been reported (Marubayashi et al., 2010; Harry et al., 2012; Kalkat et al., 2017; Johnson et al., 2018). Recently, gain-of-function (GOF) mutations in STAT3 have been observed in patients with leukemia and lymphoma, and the most common site for these somatic mutations occurs in the Src homology 2 (SH2) domain, highlighting the importance of STAT3 as a valuable target in hematologic cancers (Klein et al., 2021). The results of a study revealed that during the last reprogramming phase of the pre-induced pluripotent stem cells (pre-iPSCs), JAK/STAT3 activity plays a key role in promoting the pluripotency establishment at the epigenetic level through open-chromatin formation and facilitation of DNA demethylation/*de novo* methylation. However, the exact role of the epigenetic mechanism involved in STAT3 activation has not yet been elucidated (Tang et al., 2012). In this review, we will first examine the importance of the STAT3 signaling pathway in hematologic cancers, and then summarize the epigenetic variations affecting the JAK-STAT signaling pathway. We will also describe other epigenetic-associated proteins such as p66a (GATAD2A) and the significance of targeting the JAK-STAT signaling pathway in leukemia treatment.

## STAT Signaling

The discovery of the JAK/STAT pathway happened through a series of investigations looking into the relationship between interferon responses and signal transduction (Velazquez et al., 1992). The STAT family includes seven members: STAT1, STAT2, STAT3, STAT4, STAT5 (a/b), and STAT6 (Subramaniam et al., 2013; Rezapour et al., 2019). There is a standard structural pattern in all seven STAT proteins (Figure 1). JAK proteins have seven conserved JAK homology (JH) domains ranging from 120 to 140kDa. The JAK kinase C terminal contains two JH tyrosine catalytic (JH1) domains along with a pseudokinase domain (JH2). The SH2-like domain that contains JH3–JH5 acts as a connector of the C-terminal and N-terminal domains (Pencik et al., 2016). STAT-activated proteins interact with one another *via* their SH2 domains to form homo- or hetero-dimers, which then move into the nucleus to activate target gene transcription (Liu et al., 2018). The gene coding STAT3 is located on the chromosome 17 (17q21.1; Rezapour et al., 2019) and consists of four isoforms: STAT3α, STAT3β, STAT3γ, and STAT3δ (Aigner et al., 2019). STAT3α with a molecular weight of ~92kDa is the most frequent structure, containing domains of ND, CCD, DBD, linker, SH2, and transcriptional activation domain (TAD), and predominantly associated with cell proliferation and transformation (Shi et al., 2018). A variety of mechanisms including JAK/STAT3, Ras/mitogen-activated protein kinase (MAPK), and non-receptor tyrosine kinase (NTRK) signaling pathways enable STAT3 activation (Groner et al., 2008). The protein inhibitors of activated STATs (PIAS) adversely control STAT signaling. PIAS regulates and restricts STAT signaling by either intervening in the DNA-binding action of STATs or *via* an E3 ligase of a small ubiquitin-like modifier (SUMO) which induces STAT proteolysis. Meanwhile, cytokine signaling silencer (SOCS) proteins limit JAK/STAT signals by restraining the activity of JAK kinases and challenging interlinkage with STATs.

**Figure 1:** The structure of signal transducer and activator of transcription (STAT) family. A full-length stat consists of N-Terminal domain (required for STAT oligomerization and stabilization on DNA), Coiled-Coiled domain (needed as a nuclear localization signal for stimulation), DNA binding domain (binds DNA elements), linker domain, src homology 2 domain (SH2: mediated homo or heterodimer formation, bind transcriptional activation domain of adjacent STAT monomer), and C-terminal transcriptional activation domain (TAD: Y and S within the C-terminal are the phosphorylation sites).

STAT3 is a key downstream signaling mediator of gp130, a receptor previously revealed to activate the HSCs’ self-renewal (Kleppe et al., 2017). The induction of STAT3 proteins markedly contributes to the generation of mature hematopoietic cells by affecting cellular growth, survival, and lineage specificity. For instance, conditional JAK1 deletion, a principal mediator of STAT3 activation in HSCs, potently reduces HSCs’ self-renewal regeneration and modifies lympho-myeloid differentiation *in vivo* (Kleppe et al., 2017). Despite the role of STAT3 in hematopoietic cell proliferation, survival, and differentiation, its participation in leukemogenesis has not yet been elucidated. The constitutive stimulation of STAT3 has extensively been documented in both acute and chronic leukemias. Indeed, it seems that dysregulated STAT3 stimulation may arise from the hyperactivation or overexpression of cellular oncogenic tyrosine kinases or leukemic fusion oncoproteins (Dorritie et al., 2014). Meanwhile, granulocyte colony-stimulating factor (G-CSF) stimulates the induction of STAT3α to improve acute myeloid leukemia (AML) cell line proliferation and regulates CK2 protein kinase, the transcription of the Forkhead box O3 (FOXO3a) gene, by inducing STAT3 through JAK/STAT3 and PI3K/AKT/mTOR signaling axis, leading to leukemia stem cells growth (Shi et al., 2018). Furthermore, STAT3 activation through JAK/STAT3 and Ras/Raf/MAPK has been reported in an *in vitro* study conducted on the K562 chronic myeloid leukemia (CML) cell line (Shi et al., 2018). Besides, the study of STAT3 mutations in patients with large granular lymphocytic (LGL) leukemia showed that the mutations in STAT3 introduced an amino acid replacement in the encoded protein (Koskela et al., 2012). In another study on T-LGL patients, it was found that all mutations were missense mutations, and Tyr640Phe and Asp661Tyr were reported as the most-shared mutations in these patients. Surprisingly, some STATs can repress the transcription of their target genes (Kang et al., 2013; Saraei et al., 2019). Signaling *via* the JAK/STAT pathway is a well-organized mechanism in normal tissues controlling various stages of cell development (Li et al., 2016). Initially, STAT proteins have been identified as latent transcription factors in the cytoplasm (Zhang et al., 2016). Each member of the STAT family has a unique function. For example, STAT3 and STAT5 contribute to cancer progression, while STAT1 can suppress it. Continuous activation of STAT3/5 results in a reinforcement of chronic inflammation and thus increases healthy cells’ sensitivity to cancer. Some cytokines, including IL-12, IL-4/IL-13, and IFN-α activate STAT2, STAT4, and STAT6 (Rani and Murphy, 2016). Therefore, not all STAT proteins are exclusively involved in inflammation and malignancy growth (Wong et al., 2017). STAT3 and STAT5 can regulate the development of specific cancer cells, such as the cells with a BCR-ABL1 fusion protein (Coffer et al., 2000; Shomali et al., 2020). Various mechanisms of carcinogenesis, including the induction of the cell cycle, apoptosis, angiogenesis, metastases, and invasion are indirectly regulated by STAT3 (Loh et al., 2019). Numerous cytokines and growth factors can activate STAT3 and STAT5a/b, including interleukin (IL)-6, epidermal growth factor (EGF), platelet-derived growth factor (PDGF), hepatocyte growth factor (HGF), and insulin-like growth factor (IGF; Kim et al., 2018). Once the molecules are attached to their specific receptors on cell surface membranes, JAK kinases are activated and subsequently trigger the phosphorylation of tyrosine residues on receptors that recruit STAT protein SH2 domains (Xue et al., 2002). IL-6 can activate STAT3 *via* IL-6 receptors, gp130, and JAKs (Liu et al., 2010). Dimerization of the gp130 receptor occurs when IL-6 is bound to its receptor, which allows JAK to be active due to its interaction with gp130. Then, tyrosine residue phosphorylation is triggered on gp130, providing docking positions to inert STAT3 monomers, causing the phosphorylation of Tyr705 residues of STAT3 (Hirano et al., 2000). STAT3-activated monomers are dimerized by binding to the phosphorylated residue of the Tyr705 portion of the STAT monomer to the SH2 space of another STAT monomer (Haura et al., 2005). Nuclear translocation occurs immediately with the intervention of importin alpha5 (NPI-1; Ma and Cao, 2006). STAT3 dimers are connected to the STAT3-specific DNA-response elements of the target, allowing them to be transcribed (Figure 2; Jing and Tweardy, 2005; Loh et al., 2019). Besides, the STAT family participates with other transcription factors, including RUNX family proteins, nuclear factor-kappa B (NF-κB), and p53 (Loh et al., 2019; Shomali et al., 2021).

**Figure 2:** The binding of different ligands to their receptors on the cell surface allows the STAT to be phosphorylated inside the cell and thus transferred to the nucleus for binding the target gene to the promoter region, activating transcription. It regulates cell proliferation and survival by controlling Cyclin D1, cMyc, BclXL, Mcl1, and p5, and also is involved in cell migration *via* the control of Rho and Rac. STAT also regulates the angiogenesis required for tumor growth and metastases *via* VEGF and HIF5-007.

STAT3 has been considered a potential therapeutic objective for cancer for several reasons. First, it is stimulated in a broad range of malignancies, and its *in vitro* inhibition leads to growth arrest and apoptosis in human cancer models. Second, different carcinogenic pathways converge in STAT3 and concurrently inhibit several upstream tyrosine kinases (Wong et al., 2017).

## Epigenetic Regulation Mechanism

Epigenetic regulation is a central property of eukaryotic genomes (Feschotte and Pritham, 2007), which alters gene expression without altering the DNA sequence (Jaenisch and Bird, 2003). Epigenetic processes include DNA methylation, histone modifications, small RNAs, and protein-protein interactions (Cheng et al., 2019; Alizadeh et al., 2020). It has been indicated that atypical epigenetic modulation of gene expression is related to both hematological (Mercurio et al., 2010) and solid malignancies (Vendetti and Rudin, 2013; Nabipoorashrafi et al., 2020). In comparison to genetic mutations, the potential to reconstruct the epigenetic site in the epigenome of malignant development and the production of next-generation “epidrug” is one of the most promising objective therapies for the diagnosis, prognosis, and treatment of cancers (Nebbioso et al., 2018), as well as preventing and reversing the drug resistance (Miranda Furtado et al., 2019). DNA methylation plays an important function in the epigenetic regulation of oncogenes expression (Easwaran et al., 2014). Approximately 60–80% of CpGs in the human genome are methylated in healthy cells (Laan et al., 2020). DNA methylation in mammalian cells is limited to CpG regions that usually occur in promoter areas and thereby prevents gene transcription, while gene activation is exerted by its demethylation (Figure 3; Kong et al., 2019). The methylation of the promoter area allows the regulation of differential gene expressions, and may also be involved in chronic lymphoblastic leukemia (CLL) pathogenesis (Andreani et al., 2020). The DNA methyltransferases (DNMTs), such as DNMT1, DNMT3A, DNMT3B, and DNMT3L, can methylate DNA by passing the methyl group into the cytosine pyrimidine base in 5′-CpG-3 dinucleotides (Rajabi et al., 2016). DNMT3 is a *de novo* methyltransferase whereas DNMT1 preserves the methylation pattern fidelity of replicated daughter strands (Subramaniam et al., 2014). DNMT1 localizes to replicate foci and mostly preserve DNA methylation patterns from template strands to new DNA strands (Rajabi et al., 2016). DNMT1 can perform *de novo* methyltransferase activity through DNMT3a and DNMT3b during development (Ko et al., 2005). Notably, DNMT1, DNMT3a, and DNMT3b are usually overexpressed in cancer cells (Qu et al., 2010), and DNMT1 and DNMT3b are essential for silencing the genes in human cancer cells (Rajabi et al., 2016). Currently, DNA methyltransferase inhibitors (DNMTi) are commonly used to restore misplaced forms of DNA methylation in cancer cells (Maes et al., 2013; De Smedt et al., 2018; Akbari et al., 2020).

**Figure 3:** Methylation and its function in the genome of healthy and cancer cells. Cytosine methylation in cells is regulated by DNA methyltransferases (DNMTs). By switching methyl groups from S-adenosylmethionine (SAM) to S-adenosylhomocysteine (SAH), methylation is done in the CPG Islands in the promoter of genes. Normal cell promoters are immune to methylation, resulting in gene transcription. However, in mutant and cancerous cells in the promoter regions of the genes, hypermethylation is done and inhibits the transcription of such genes, such as tumor suppressor genes, as a result of gene silencing.

## The Function of JAK/STAT Signaling in Hematopoietic Malignancy

Normal hematopoietic cells are differentiated and matured by cytokines. However, leukemia cells are characterized by a lack of differentiation. Although the activity of STAT3 in normal cells is rapid and transient, aberrant expression of STAT3 activity always occurs in leukemic cells, which in turn, provokes the proliferation of leukemic cells, and prevents differentiation and apoptosis (Schemionek et al., 2012). Based on molecular analysis, G-CSF triggers STAT3α activation to enable the proliferation of AML cell lines. Also, STAT3 can be activated through the JAK/STAT3 and Ras/Raf/MAPK pathways, which start Forkhead box M1 (FOXM1) gene transcription and stimulate CML cells proliferation *in vitro* (Mencalha et al., 2012). In detail, G-CSF binding to its ligand on the cell surface results in the Y705 domain phosphorylation in STAT3. Finally, multi-signal transduction pathways are activated *via* Ras/Raf/MAPK, PI3K, and JAK/STAT cascades (Ward et al., 1999). Remarkably, the STAT3 protein controls G-CSFR-mediated signaling pathways and obstructs the differentiation of granulocytes (Hillmer et al., 2016). In this regard, scientists have shown that STAT3 inhibition is effective in hampering the proliferation and survival of leukemia cells (Wu et al., 2015). The role of STAT3 in apoptosis is also remarkable as activated STAT3 stimulates the expression of anti-apoptotic genes and inhibits apoptosis in leukemic cells, while its inhibition regulates the expression of proapoptotic genes, causing the apoptosis of leukemia cells (Zhou et al., 2009; Mencalha et al., 2010). Therefore, the activation status of STAT3 may be considered as a prognosis target for leukemia (Fathi et al., 2018). Moreover, it has been identified that STAT3 and STAT5 are important for hematopoietic malignancies that affect both myeloid and lymphoid compartments (Zhang et al., 2007). JAK2 mutant has been described in several cases with myeloproliferative neoplasms (MPNs) polycythemia Vera, thrombocythemia, myelofibrosis, and also a high level of STAT3 has been detected in special ovarian cancer cell lines (Nowak et al., 2017).

Evidence suggest that deregulated STAT3 activity leads to increased drug resistance in leukemia and lymphoma. Therefore, it is important to develop drug molecules based on the chosen STAT3 target in hematological neoplasms (Brachet-Botineau et al., 2020).

### STAT3 in Acute Lymphoblastic Leukemia and CLL

Although the role of STAT3 in ALL has not been well determined, pieces of evidence highlight the potent anti-proliferative and anti-tumor inhibition of STAT3 in B-ALL cells in clinical studies (Belton et al., 2016). It is known that phosphorylation of STAT3 on S^727^ is a signature of CLL development (Hazan-Halevy et al., 2010), as it can regulate the transcription function of the STAT3, and is associated with mitochondrial localization of STAT3 in CLL patients’ cells (Brachet-Botineau et al., 2020).

### STAT3 in T-LGL Leukemia

In 40% of patients with leukemia-LGL, an unusual T-cell disease, STAT3 mutations have been identified. STAT3 mutations are rare in patients with lymphoid neoplasms and are found in 1.6% of T-cell neoplasms patients and 2.5% of patients with diffuse large B-cell lymphoma (Couronné et al., 2013). Furthermore, mutations in the STAT3 SH2 domain (Y640F, D661Y/V) have also been identified in T-LGL leukemia (Rajala et al., 2014).

### STAT3 in Hodgkin Lymphoma and Non-hodgkin Lymphoma

Studies have shown the importance of upregulated STAT3 in the proliferation and survival of Hodgkin’s cells (Kube et al., 2001). Holtick et al. (2005) described that STAT3 is essential for the proliferation of HL cells and is the target of Tyrphostin AG17, which confers apoptosis sensitization. Anaplastic large cell lymphoma (ALCL) may be classified into positive and negative subgroups of anaplastic lymphoma kinase (ALK), depending on rearrangements of the ALK genes. The fusion protein NPM-ALK is the main oncogenic catalyst in ALK+ ALCL and it activates STAT3 (Zamo et al., 2002; Brachet-Botineau et al., 2020). It has been shown that dysregulation of the STAT3 function contributes to the pathogenesis of cutaneous T-cell lymphoma (CTCL) and the progression of cancer (Netchiporouk et al., 2014). Patients with adult T cell leukemia/lymphoma (ATLL) have been shown to have active mutations in Y640F and D661Y/V/H/N in the STAT3 SH2 domain, leading to increased STAT3 phosphorylation and cell growth (Kücük et al., 2015; Brachet-Botineau et al., 2020). Moreover, in patients with NK/T cell lymphoma, increased phosphorylation and STAT3 transcriptional activity have been observed due to active E616 G and E616 K mutations in the SH2 domain (Song et al., 2018).

## The Role of Methylated SOCS in the JAK/STAT Pathway

Suppressor of cytokine signaling plays a key role in the proteins as negative regulators of Jak-STAT signaling (Subramaniam et al., 2013). The SOCS family involves eight members including SOCS1-7 and CIS, all of which have a main Src-homology 2 domain (SH2) and a conserved C-terminal domain known as the SOCS box (Chim et al., 2004). They are involved in several inflammatory disorders and tumors, including hepatocellular carcinoma, breast cancer, colorectal, and cervical cancer. Dysregulation of the SOCS genes has been detected in solid tumors as well as hematological malignancies including myeloproliferative disorders and AML with unfavorable prognoses. SOCS5 is a tumor suppressor gene that controls the EGFR and JAK/STAT signal pathways negatively. Also, JAK/STAT pathway is negatively regulated by SOCS1 and Src homology region 2 domain-containing phosphatase-1 (SHP-1; Chim et al., 2004). SHP1 is a negative signaling pathway for JAKs, which is activated in MPNs and leukemia (Yang et al., 2015). Sharma et al. (2019) have shown that SOCS5 is epigenetically regulated by DNA methylation and histone deacetylation. They also demonstrated that SOCS5 silencing substantially improved the proliferation of T-ALL *in vitro* and a murine model of human leukemia. They have shown that SOCS1 is rarely inactivated by methylation. On the other hand, it has been shown that SHP1 is frequently silenced by methylation in leukemia and lymphomas, and SHP1 methylation was involved in the constitutive activation of STAT3. They suggested that SHP1 methylation may be an effective epigenetic factor that correlates with SOCS6 and enhances neoplastic cell growth (Sharma et al., 2019). Moreover, silencing of DNMT1 hinders the initiation of the JAK2/STAT3 pathway in lipopolysaccharide- (LPS-) stimulated RAW 264.7 macrophage cell line. Cheng et al. (2014) showed that hypermethylation of SOCS1 by DNMT1 causes loss of SOCS1 function in negative regulation of the JAK2/STAT3 pathway and increases the release of inflammatory cytokines induced by LPS such as interleukin-2 and TNF in macrophages. Thus, LPS can increase SOCS1 methylation by the upregulated expression of DNMT1, which leads to an inflammatory secretion of cytokines by RAW264.7 cells (Cheng et al., 2014). Moreover, SOCS proteins minimized cytokine-induced functions *via* JAK/STAT pathway, and a decreased expression of SOCS proteins resulted in increased cytokine-induced reactions to osteoarthritis (de Andrés et al., 2011). SOCS gene methylation has also been related to gene silence and increased STAT activity in ovarian and breast carcinogenic diseases (Sutherland et al., 2004). Other investigations have revealed that the levels of SOCS5 mRNA were related to its promoter methylation, and the IL-7R signaling pathway is negatively regulated by SOCS5 in T-ALL cells (Sharma et al., 2019). Moreover, observations signified that increased leukemia cell proliferation may rely on SOCS5 inactivation (Sharma et al., 2019). In another study, Hajime Isomoto and his coworkers found that STAT-3 was activated by IL-6 through methylation of the CPG islands in the SOCS-3 gene promoter and its shutdown. As a result, the activation of STAT3 decreased with the re-expression of SOCS3 which may be significant in the epigenetic treatment of cancer by restoring SOCS3 (Isomoto et al., 2007).

### Relation Between STAT3 and Epigenetics in Leukemia

STAT3 activation is not well-known in epigenetic processes. Reports have suggested that the activity of JAK/STAT3 plays a key role in fostering epigenetic pluripotency, *via* facilitating DNA *de novo* methylation and the formation of chromatin free during late reprogramming (Tang et al., 2012). The phosphorylated and activated STAT3 is translocated into the nucleus and increases the transcription of other oncogenes in cancerous cells. However, unphosphorylated STAT3 may also trigger gene expression *via* IL-6-based activation (Nowak et al., 2017). Xin et al. (2017) have identified a protein called P66 as an epigenetic-related protein that suppresses the transcription of new proteins through STAT3 in functional MDSCs. The P66 regulates phosphorylation and ubiquitination of STAT3 and can suppress its function through posttranslational modification. This may be a new mechanism that controls STAT3 activity in differentiating myeloid cells (Xin et al., 2017). The most common phosphorylation site associated with STAT3 activation is tyrosine phosphor-STAT3 (Y705; Diao et al., 2015). Studies have shown that p66 interacts with STAT3 and suppresses Y705-site phosphorylation, suggesting the essential role of p66 in the STAT3 activation system (Vasquez-Dunddel et al., 2013).

DNA methylation in acute myelogenous leukemogenesis is a subject that has widely been used in clinical studies and has become a diagnostic, prognostic, and potential therapeutic target for AML. Also, a further understanding of the relationship between DNA methylation, genetic anomalies, and gene expression may provide exceptional experiences in the pathogenesis of AML (Xin et al., 2017). As discussed above, SHP1 is the negative signaling pathway for JAKs and is activated in MPN and leukemia, and Hypermethylation of SHP1 has been observed commonly in AML patient samples and leukemia characterized by *t*(8;21) or inv(16), was shown by samples of hypermethylated SHP1. Hypermethylated SHP1 was found in 17% of T-ALL and 11% of B-ALL samples (Ghoshal Gupta et al., 2008). Similarly, SOCS1 hypermethylation was reported among AML patients especially among those with *t*(15;17; acute promyelocytic leukemia; Chen et al., 2003). Other pieces of evidence confirmed abnormal hypermethylation of SHP1 in different leukemic cell lines and mononuclear bone marrow patients with MPNs (Yang et al., 2015). Drennan et al. (2017) also identified a strong connection between IL-10 production and locus methylation status, including an area with STAT3 site, implying that B10 functionality is epigenetic programming in CLL. Previous studies have shown STAT3 activation *via* BCR-ABL, JAK2V617F, and KITD816V in mice (Coppo et al., 2006). Epigenetic dysregulation in MDS and AML is an early event of somatic mutations in hematopoietic stem cells which cause a potential deficit in protein level and a poor prognosis. In CLL, epigenetic controllers are rarely mutated, but very deregulated with a reduced appearance in connection with disease progression (Bagacean et al., 2018).

### Relation Between STAT3 and Epigenetics in Non-leukemic Hematologic Malignancies

Epigenetic factors play an important role in the pathogenesis of autoimmune systemic lupus erythematosus (SLE). For example, RFX1, which is a transcriptional control factor, regulates the expression of the target gene by binding to the X-box in the DNA sequence. Studies have shown that STAT3 phosphorylation by IL-6 suppresses RFX1 expression in CD4+ T cells in patients with SLE, and the pSTAT3 level was high in CD4+ T cells among SLE cases (Zhao et al., 2018). In multiple myeloma, CD38 expression is affected by IL-6, and since IL-6 can activate various signaling pathways, including STAT3, STAT3 is considered the strongest negative CD38 regulator. The results of the studies have evidenced that STAT3 is an important factor in the expression of CD38 in MM cells in the BM environment. These outcomes may introduce new combination therapy options by targeting CD38 with a JAK-STAT pathway inhibitor (Ogiya et al., 2020; Shomali et al., 2021).

## Epigenetic Therapy in Hematological Malignancies

Given the impact of the JAK/STAT pathway on cancer growth and development, targeting this pathway as a cancer treatment is a good choice. There are many strategies for targeting STAT proteins. Since STAT3 and STAT5 are more involved in several malignancies, more studies have been done to regulate them (Furqan et al., 2013). Additional research has been done to create JAK/STAT pathway inhibitors, then several of these pathway inhibitors are being studied in leukemia clinical trials (Buchert et al., 2016). Ruxolitinib and Tofacitinib are two effective JAK inhibitors. Ruxolitinib targets JAK1 and JAK2, while Tofacitinib targets JAK1, JAK2, and JAK3 (Flanagan et al., 2010; Stover et al., 2018). Moreover, OPB-31121 is a small regulatory molecule that is engineered to bind to the SH2 domain of STAT3/5 and prevents its downstream processes (Brambilla et al., 2015; Pencik et al., 2016; Brachet-Botineau et al., 2020). AZD9150 is also a 16-oligonucleotide molecule that attaches to untranslated mRNA STAT3 regions and prevents the translation of STAT3 protein (Reilley et al., 2018). Only a few inhibitors, including AZD9150 and OPB-3112, have passed phase I clinical trials for leukemia (Pencik et al., 2016). There are drugs designed to suppress other kinases but they also have an inhibitory effect on the JAK group. For instance, Lestaurtinib (CEP-701) is an FLT3 and TrkA inhibitor, but it has also been reported to inhibit JAK and may also be used to treat AML (Hexner et al., 2008). Qin JJ et al. argued that there are new ways to induce STAT3 protein breakdown through PROTAC or STAT3 binding inhibition that need to be investigated, which could lead to the discovery of more effective treatment and prevention methods (Figure 3; Qin et al., 2019).

It is noteworthy that the alteration of epigenetic pathways can also play a role in cancer initiation and progression. Several compounds have been developed to target epigenetic enzymes for epigenetic therapy in hematological malignancies and solid tumors. As a consequence, epigenetic expansion and increased resistance to epidrug therapy are possible factors of combination therapy (Kerry et al., 2017). The activation and/or repression of epigenetics can result in the suppression of tumor growth or sensitization to anticancer therapies. It is now well-established that epigenetically silenced genes can be reactivated by the action of small molecules, epidrugs, capable of correcting epigenetic defects pharmacologically. Epidrug therapy can reactivate silent gene transcription, suppress enzymes such as DNMTs or HDACs, and restitute natural cell growth and differentiation (Carafa et al., 2013). Targeting epigenetic aberrations is a well-known strategy for treating patients with AML, and several epigenetic drugs have been clinically approved which affect different stages of cell development (Mehdipour et al., 2015). AML clinical trials have recently tested the effectiveness of DNMTi such as 5-AZA and decitabine, and HDAC inhibitors, such as SAHA, Romidepsin, and LBH589. Currently, these epidrugs are under clinical study individually or in conjunction with other medical therapies for hematological malignancies (Figure 4; Nebbioso et al., 2015).

**Figure 4:** Scheme of STAT3 function and epigenetic changes in cancers and current pharmaceutical drugs that target epigenetic mechanisms (DNMT1) and STAT signaling pathway inhibitors.

## Conclusion

The detection of genetic mutations in specific enzymes involved in epigenetic regulation is invaluable. As discussed above, STAT3 has a bilateral function, resulting in both embryonic developmental activity and oncogenic function. Due to the overexpression of STAT3 in malignancies that leads to tumor progression, STAT3 is considered a therapeutic target. Importantly, the identification of new STAT3 inhibitors for the treatment of certain leukemias is of paramount importance. To sum up, we suggest that developing inhibitors that affect the JAK/STAT signaling pathway in cancer cells through various pathways, such as phosphorylation in serine and tyrosine residues, acetylation, methylation, and glycosylation may be a potential therapeutic strategy for a variety of hematological malignancies.

## Author Contributions

EZ, AY, HR, FM, NS, HK, SS, MS-D, and SV-S took part in conceptualization and also drafted the main text, figures and tables. AY drew the figures. FM, AY, and NS participated in the writing and scientific editing of the manuscript. MJ and MF supervised the work and provided the comments and additional scientific information. All authors read and approved the final version of work to be published.

## Conflict of Interest

The authors declare that the research was conducted in the absence of any commercial or financial relationships that could be construed as a potential conflict of interest.

## Publisher’s Note

All claims expressed in this article are solely those of the authors and do not necessarily represent those of their affiliated organizations, or those of the publisher, the editors and the reviewers. Any product that may be evaluated in this article, or claim that may be made by its manufacturer, is not guaranteed or endorsed by the publisher.
